The article "Genetic Polymorphism of Interferon Regulatory Factor 5 (IRF5) Correlates with Allograft Acute Rejection of Liver Transplantation" was retracted in 2019. Reasons: missing or withdrawn patient consent; ethical violations by an author; concerns about the data.

# Genetic Polymorphism of Interferon Regulatory Factor 5 (IRF5) Correlates with Allograft Acute Rejection of Liver Transplantation

**DOI:** 10.1371/journal.pone.0094426

**Published:** 2014-04-30

**Authors:** Xiaobo Yu, Bajin Wei, Yifan Dai, Min Zhang, Jian Wu, Xiao Xu, Guoping Jiang, Shusen Zheng, Lin Zhou

**Affiliations:** 1 Key Lab of Combined Multi-Organ Transplantation, Ministry of Public Health, the First Affiliated Hospital, School of Medicine, Zhejiang University, Hangzhou, Zhejiang, China; 2 Division of Hepatobiliary and Pancreatic Surgery, Department of Surgery, the First Affiliated Hospital, School of Medicine, Zhejiang University, Hangzhou, Zhejiang, China; Penn State University, United States of America

## Abstract

**Background:**

Although liver transplantation is one of the most efficient curative therapies of end stage liver diseases, recipients may suffer liver graft loss opst-operation. IRF-5, a member of Interferon Regulatory Factors, functions as a key regulator in TLR4 cascade, and is capable of inducing inflammatory cytokines. Although TLR4 has been proved to contribute to acute allograft rejection, including after liver transplantation, the correlation between IRF5 gene and acute rejection has not been elucidated yet.

**Methods:**

The study enrolled a total of 289 recipients, including 39 females and 250 males, and 39 recipients developed acute allograft rejection within 6 months post-transplantation. The allograft rejections were diagnosed by liver biopsies. Genome DNA of recipients was extracted from pre-operative peripheral blood. Genotyping of IRF-5, including rs3757385, rs752637 and rs11761199, was performed, followed by SNP frequency and Hardy-Weinberg equilibrium analysis.

**Results:**

The genetic polymorphism of rs3757385 was found associated with acute rejection. G/G homozygous individuals were at higher risk of acute rejection, with a *P* value of 0.042 (OR = 2.34 (1.07–5.10)).

**Conclusions:**

IRF5, which transcriptionally activates inflammatory cytokines, is genetically associated with acute rejection and might function as a risk factor for acute rejection of liver transplantations.

## Introduction

Liver transplantation has been accepted worldwide as an efficient way of treating end stage liver diseases and acute liver failure. Immune system elicits complex and aggressive reaction post-transplantation, which even destroys the graft [1], [2]. Although the total incidence of allograft rejection decreases dramatically due to immunosuppressive therapies [3], acute rejection episodes still occur among 15–45% recipients within several months, which leads to higher incidence of chronic organ dysfunction and suboptimal long-term outcomes [3].

The article "Genetic Polymorphism of Interferon Regulatory Factor 5 (IRF5) Correlates with Allograft Acute Rejection of Liver Transplantation" was retracted in 2019. Reasons: missing or withdrawn patient consent; ethical violations by an author; concerns about the data.

For years, acute rejection was considered as response of adaptive immune system. However, it is gradually accepted that, by responding to the released danger signal, innate immune reaction also functions as a pivotal trigger in acute rejection [4]. Toll-like Receptors (TLR), which recognize pathogen-associated molecular patterns (PAMP) on microorganisms in innate immune response, are now proved to initiate inflammation by recognizing molecules released from damaged cells during organ transplantation [5], [6], and prevent graft tolerance in dependence of type I IFNs [7]. Nevertheless, TLRs pathway can also induce immunosuppression [8], [9], and we also confirmed the contribution of TLR4 to liver graft rejection [10]. Therefore, regardless of enhanced alloimmune response or immunosuppression, the elucidation of TLR signal pathway in acute rejection, especially TLR4, is urgently needed.

Interferon Regulatory Factors (IRFs), including nine family members, play important roles in TLRs signal cascade [11], [12]. Each contains a DNA-binding domain recognizing IFN-Stimulated Response Element (ISRE), which locates upstream of interferon genes [13]. Thus IRFs could involve in regulating the innate immune reaction and immune cell development through transcriptional activation of type I IFNs and other proinflammatory cytokines [14]–[16]. Studies on gene expression profiling in acute rejection also indicated the association between acute allograft rejection and IRFs, such as IRF9, IRF3 and IRF5 [17]–[19].

As a key regulator of TLR4 cascade in innate immune responses, IRF5 can activate the transcription of type I IFNs when it forms homodimers or heterodimers with IRF3, or suppress them via interacting with IRF7 [14], [20]. Moreover, IRF5 is also responsible for the production of inflammatory cytokines, such as IL-6 and TNF-α [20], [21]. Several studies also associated IRF5 with higher risk of systemic lupus erythematosus (SLE) [22], [23], while some other SNPs of IRF5 are proved responsible for a lower risk of its development [24], [25]. Researchers further found IRF5 to be critical for IFN-α secretion by dendritic cells in SLE patients [26]. Other genetic studies confirmed its association with rheumatoid arthritis (RA) in different populations [27]–[29].

Although there has been no direct evidence for the involvement of IRF5 in acute allograft rejection, the fact that IRF5 transcriptionally activates IFNs and other pro-inflammatory genes in cell apoptosis and T cell activation, and functions as a key factor of TLR4 cascade [26], [30], suggests that it is reasonable to perform association studies on acute rejection. Thus understanding of how IRFs participate will help us with the development of treatment of acute rejection. Meanwhile, genetic association studies provide correlation between disease status and genetic variation, such as SNPs and haplotypes that contribute to the disease, and therefore could facilitate identification of new biomarkers for risk prediction and prognosis.

The article "Genetic Polymorphism of Interferon Regulatory Factor 5 (IRF5) Correlates with Allograft Acute Rejection of Liver Transplantation" was retracted in 2019. Reasons: missing or withdrawn patient consent; ethical violations by an author; concerns about the data.

Three SNPs of IRF5 gene were involved in this study, including rs3757385, rs752637 and rs11761199, and among them rs3757385 and/or rs752637 had been found to be associated with SLE and RA [29], [31]. Our new findings suggested that rs3757385 might be a genetic marker for acute rejection prognosis, and the biological function of IRF5 as well as other IRFs in acute allograft rejection will be worth studying.

## Methods

### Population

A total of 289 recipients who received their liver grafts during 2006 to 2011, including 250 males and 39 females, were enrolled in this association study. Those diagnosed with drug-induced hepatitis, autoimmune hepatitis and sclerosing cholangitis were excluded. Moreover, we excluded patients that underwent a second or subsequent liver transplantation or multiple organ transplantation. Data of age, gender and primary diagnoses were collected for population study. All the recipients followed a unique triple combination of immunosuppressive regimen, including tacrolimus, corticosteroid and mycophenolate mofetil. In brief, the minimum level of tacrolimus blood concentration was maintained at 10–12 ng/ml for the first month after transplant, 8–10 ng/ml later in the first year, and 5–8 ng/ml thereafter. Mycophenolate mofetil was administered 1–2 g per day. Corticosteroid treatment was initiated with 1000 mg prednisolone once during the operation, continued with administration of gradually reduced meth-prednisolone starting at 240 mg on day 1 and ending up at 2.5 mg before discontinuation after 2 months [32]. Among the recipients, 39 finally developed acute rejection.

### Definition of acute rejection

The diagnoses of acute rejection were confirmed by liver biopsy and graded by Banff schema. Rejection occurred within 6 months was considered as acute rejection [33], [34].

### Ethics statement

Written informed consents were obtained, and for children, they were obtained from the next of kin. The research procedure was approved and supervised by the Ethical Review Committee of the First Affiliated Hospital, School of Medicine, Zhejiang University, and we followed the World Medical Association's Declaration of Helsinki.

### DNA extraction and genotyping

Peripheral blood genomic DNA was extracted for genotyping. Based on the data of Hapmap (http://www.hapmap.org), we selected candidate SNPs of IRF5 in accordance with the rule that minor allele frequency and r^2^ should be no less than 20% and 0.8. The genotyping was performed by SNaPshot (Applied Biosystems, CA), followed by data collection and generation from ABI3130xl Genetic Analyzer (Applied Biosystems, CA) and GeneMapper 4.0 (Applied Biosystems, CA), respectively.

The article "Genetic Polymorphism of Interferon Regulatory Factor 5 (IRF5) Correlates with Allograft Acute Rejection of Liver Transplantation" was retracted in 2019. Reasons: missing or withdrawn patient consent; ethical violations by an author; concerns about the data.

### Association analysis

Genetic association between SNPs or haplotypes and acute rejection was analyzed by SNPStats (http://bioinfo.iconcologia.net/snpstats) or Haploview (http://www.broad.mit.edu/mpg/haploview).

### IRF5 mRNA expression assay

Total RNA was extracted from peripheral blood mononuclear cells of recipients within 6 months post-transplant, and cDNA was synthesized by reverse transcription kit (Bio-Rad, CA). The expression of IRF5 was detected on ABI 7500 Fast Real-Time PCR System (Applied Biosystems, CA) using iTaq Universal SYBR Green Supermix real-time PCR kit (Bio-Rad, CA). The primer pairs of IRF5 and GAPDH for real-time PCR detection were listed as following; IRF5, forward 5′- GACATCCCCAGTGACAAGCA -3′, reverse 5′- AGAACACCTTGCACTGACACA -3′, and GAPDH, forward 5′-ATGGGGAAGGTGAAGGTCG-3′, reverse 5′-GGGGTCATTGATGGCAACAATA-3′. The real-time PCR procedure included a cDNA denaturation at 95°C for 20 sec, and then 40 cycles of amplification with 10 sec at 95°C and 30 sec at 58°C, following with a melt-curve analysis. The relative expression of IRF5 mRNA was calculated by ΔΔCT method.

### Statistic analysis

For clinical relevance of primary diagnoses and acute rejection, Fisher's exact test was performed with Graphpad Prism 6.0 (Graphpad Software, CA). For survival analysis, cumulative graft rejection rate was estimated using the Kaplan-Meier method. The relationship between risk of acute rejection and genotypes was examined using the log-rank test with Graphpad Prism. For analysis of IRF5 mRNA expression, unpaired t-test or one-way ANOVA test was used for comparison of two groups or more than two groups with Graphpad Prism. A two-tailed *P* value less than 0.05 was considered statistically significant.

## Results

A cohort of 289 recipients was enrolled in the association study. We first analyzed the clinical data from individuals, and no statistical significance was found among age, gender, Model For End-Stage Liver Disease (MELD) score and most of the primary diagnoses, except Hepatitis B Virus (HBV) infection (Table 1). We found HBV infection to be one of the risk factors for acute liver graft rejection, and recipients with HBV infection were at higher risk of rejection. Moreover, our genetic association analysis indicated that the incidence of acute rejection in G/G homozygtes of rs3757385 was relatively higher (Table 2). Linkage disequilibrium analysis showed that haplotypes could be formed by rs3757385 and rs752637 (Figure 1), yet no association was found between haplotype groups and acute rejection (Table 3).

The article "Genetic Polymorphism of Interferon Regulatory Factor 5 (IRF5) Correlates with Allograft Acute Rejection of Liver Transplantation" was retracted in 2019. Reasons: missing or withdrawn patient consent; ethical violations by an author; concerns about the data.

**Figure 1:** The linkage disequilibrium among 3 SNPs. 1 to 3 represented rs3757385, rs752637 and rs11761199 respectively, and rs3757385 and rs752637 formed a haplotype block by LD analysis.

**Table 1:** Characteristics and primary diagnosis of 289 liver transplantation recipients assigned to a non-rejection or acute rejection group.

	Non-rejection	Acute Rejection	*P* value
Age (year)	13–71	31–71	NA
Sex			0.6234
Male	215 (86.0%)	35 (89.7%)	
Female	35 (14.0%)	4 (10.3%)	
MELD Score			0.1945
<10	41 (16.4%)	11 (28.2%)	
10–19	94 (37.6%)	11 (28.2%)	
20–29	77 (30.8%)	9 (23.1%)	
>29	38 (15.2%)	8 (20.5%)	
Primary diagnosis			
HBV infection	148 (59.2%)	30 (76.9%)	0.0351
	102 (40.8%)	9 (23.1%)	
HCC	99 (39.6%)	15 (38.5%)	1.000
	151 (60.4%)	24 (61.5%)	
Fulminant hepatitis	49 (19.6%)	8 (20.5%)	0.8320
	201 (80.4%)	31 (79.5%)	
Decompensated liver cirrhosis	142 (56.8%)	20 (51.3%)	0.6035
	108 (43.2%)	19 (48.7%)	

MELD, model for end-stage liver disease; HCC, hepatocellular carcinoma; NA, not applicable.

**Table 2:** Association of genetic polymorphism of IRF5 with acute rejection.

SNPs of IRF5	Genetic Model	Non-rejection	Acute Rejection	OR (95% CI)	*P* value
rs3757385					
T/T	Cod	105 (42.0%)	11 (28.2%)	1.00	0.078
G/T		109 (43.6%)	17 (43.6%)	1.49 (0.67–3.33)	
G/G		36 (14.4%)	11 (28.2%)	2.92 (1.17–7.30)	
T/T	Do	105 (42.0%)	11 (28.2%)	1.00	0.096
G/T+G/G		145 (58.0%)	28 (71.8%)	1.84 (0.88–3.87)	
T/T+G/T	Re	214 (85.6%)	28 (71.8%)	1.00	0.042
G/G		36 (14.4%)	11 (28.2%)	2.34 (1.07–5.10)	
T/T+G/G	Ovd	141 (56.4%)	22 (56.4%)	1.00	1.00
G/T		109 (43.6%)	17 (43.6%)	1.00 (0.51–1.97)	
rs752637					
T/T	Cod	105 (42.0%)	12 (30.8%)	1.00	0.14
C/T		111 (44.4%)	17 (43.6%)	1.34 (0.61–2.94)	
C/C		34 (13.6%)	10 (25.6%)	2.57 (1.02–6.48)	
T/T	Do	105 (42.0%)	12 (30.8%)	1.00	0.18
C/T+C/C		145 (58.0%)	27 (69.2%)	1.63 (0.79–3.36)	
T/T+C/T	Re	216 (86.4%)	29 (74.4%)	1.00	0.067
C/C		34 (13.6%)	10 (25.6%)	2.19 (0.98–4.90)	
T/T+C/C	Ovd	139 (55.6%)	22 (56.4%)	1.00	0.92
C/T		111 (44.4%)	13 (43.6%)	0.97 (0.49–1.91)	
rs11761199					
A/A	Cod	105 (42.0%)	11 (28.2%)	1.00	0.25
A/G		111 (44.4%)	21 (53.9%)	1.81 (0.83–3.93)	
G/G		34 (13.6%)	7 (17.9%)	1.97 (0.71–5.47)	
A/A	Do	105 (42.0%)	11 (28.2%)	1.00	0.096
A/G+G/G		145 (58.0%)	28 (71.8%)	1.84 (0.88–3.87)	
A/A+A/G	Re	216 (86.4%)	32 (82.1%)	1.00	0.48
G/G		34 (13.6%)	7 (17.9%)	1.39 (0.59–3.40)	
A/A+G/G	Ovd	139 (55.6%)	18 (46.1%)	1.00	0.27
A/G		111 (44.4%)	21 (53.9%)	1.46 (0.74–2.34)	

OR, odds ratio; CI, confidence intervals.

Cod, codominant; Do, dominant; Re, recessive; Ovd, overdominant.

The article "Genetic Polymorphism of Interferon Regulatory Factor 5 (IRF5) Correlates with Allograft Acute Rejection of Liver Transplantation" was retracted in 2019. Reasons: missing or withdrawn patient consent; ethical violations by an author; concerns about the data.

**Table 3:** Association of IRF5 Haplotype with acute rejection.

SNPs combination	Non-rejection	Acute Rejection	OR (95% CI)	*P* value
rs3757385 + rs752637				
T-T	308 (61.6%)	48 (61.5%)	1.00	1.00
G-C	185 (37.0%)	28 (35.9%)	0.97 (0.59–1.60)	

Survival analysis was performed to investigate how genotypes of IRF5 influence the probability of acute rejection. In consistent with the higher risk of rs3757385 G/G homozygous recipients in acute rejection, log-rank test also indicated a predictive value of rs3757385 for rejection, instead of rs752637 and rs11761199 (Figure 2 and Table 4).

**Figure 2:** Acute rejection comparisons among SNP groups.

**Table 4:** Comparison of survival curves among SNP groups.

SNPs of IRF5	*P* value	HR (95% CI)
rs3757385		
T/T vs. G/T vs. G/G	0.075	NA
T/T vs. G/T + G/G	0.102	0.56 (0.31–1.11)
G/T vs. T/T + G/G	0.079	1.95 (0.93–4.12)
G/G vs. T/T + G/T	0.038	2.06 (1.05–5.82)
rs752637		
T/T vs. C/T vs. C/C	0.13	NA
T/T vs. C/T + C/C	0.18	0.63 (0.34–1.22)
C/T vs. T/T + C/C	0.97	0.99 (0.53–1.86)
C/C vs. T/T + C/T	0.057	1.98 (0.98–5.72)
rs11761199		
G/G vs. A/G vs. A/A	0.25	NA
G/G vs. A/A + A/G	0.46	1.36 (0.57–3.48)
A/G vs. A/A + G/G	0.26	1.43 (0.77–2.70)
A/A vs. A/G + G/G	0.098	0.56 (0.31–1.10)

HR, hazard ratio.

Since rs3757385 locates in the promoter region, we assumed that it might cause changes of IRF5 expression level. Meanwhile, IRF5 transcripts could be detected in peripheral blood mononuclear cells (PBMC) [35], which suggest a possibility to evaluate rejection by monitoring IRF5 mRNA in PBMC. Thus we compared IRF5 mRNA expression in PBMC among the different genotype groups of rs3757385, rs752637 and rs11761199 respectively. However, results from real-time PCR exhibited no significant difference among the 3 genotype groups (Figure 3).

**Figure 3:** mRNA expression level of IRF5 in PBMC. We performed real-time qPCR to detect the mRNA expression of IRF5 in the PBMC of a total of 104 recipients, of whom the rejection had not been observed within 6 months post-operation.

## Discussion

Although little direct evidence has depicted the involvement of IRF5 in acute rejection, its capability of transcriptionally activating IFNs and pro-inflammatory genes through TLR4 cascade implies potential roles. Moreover, it is genetically associated with autoimmune diseases, such as SLE and RA. Thus genetic polymorphism of IRF5 might function as a marker for risk prediction and prognosis of graft rejection. The rs3757385 SNP, locating in promoter region, participates in regulating IRF5 mRNA expression in atherosclerotic lesions [36], and affects genetic susceptibility to autoimmune diseases [29]. In this article we proved genetic polymorphism of rs3757385 to be a risk factor for acute rejection for the first time.

The article "Genetic Polymorphism of Interferon Regulatory Factor 5 (IRF5) Correlates with Allograft Acute Rejection of Liver Transplantation" was retracted in 2019. Reasons: missing or withdrawn patient consent; ethical violations by an author; concerns about the data.

Since there have been reports indicating that IRF5 mRNA expression is associated with autoimmune diseases [17], [37], in consideration of the detectability of IRF5 mRNA in PBMC [35] and genetic susceptibility of rs3757385 in acute rejection, acute rejection might be predicted by monitoring IRF5 expression. However, in this cohort, IRF5 mRNA expression level was inconsistent with rs3757385 genetic polymorphism, which could be explained from several aspects. IRF5 pre-mRNA generates alternatively spliced transcripts, but little evidence is available on how these transcripts function in physiological regulation. Thus in this study, we used the consensus sequence of IRF5 CDS for real-time analysis of the indistinguishable expression of each isoform, which suggests isoforms specific to acute rejection still need to be identified. The insignificant difference of IRFs expression may also be due to a cell-specific regulation of IRF5 mRNA by rs3757385 in immune cell subpopulations.

According to different cohort studies, MHC mismatch, T cell activity and immunosuppressive regimen, as well as age, gender, pre-LT disease, viral infection and ischemia time were involved in the outcome of graft survival. Based on our study, HBV infection could be a risk factor for acute rejection, while other studies indicated that it would decrease the incidence of acute rejection after liver transplant [38]–[40]. Therefore, if these inconsistent observations were not due to sampling bias, it might be due to the ways of preventing HBV reinfection that led to such difference. According to some studies [41]–[43], HBIG administration could benefit the recipients with better immunosuppression, and reduce acute rejection by inhibiting dendritic cells as well as provoking CD4+FoxP3+ T cells. We have developed a substitution therapy combining lamivudine (LAM) and low-dose intramuscular hepatitis B immunoglobulin (HBIG) [44], while many centers adopt a long-term regimen of high-dose administration of HBIG [40]. However, to confirm the survival benefit of HBIG for preventing postoperative HBV reinfection, further examinations and studies will be needed [45].

Genotyping of functional genes has led to improved efficacy of cancer therapy, either providing a targeted course of treatment based on their molecular designation, or avoiding harmful side effects by optimal dosing of drugs [46]. Complex diseases such as autoimmune diseases and transplantation rejections, are caused by the combination of genetic, environmental and some other factors, of which most have not been identified. The elucidation of mechanisms by which they predisposed individuals to graft rejection facilitates the application of genetic polymorphism in the development of new prognosis methods. Scientists can focus on relatively small numbers of genes which are involved in cell differentiation, proliferation and migration, and cytokine signaling, and explore their utility in personalized medicine. In the foreseeable future, personalized medicine associated with genetic information would become embedded in medical units.

The article "Genetic Polymorphism of Interferon Regulatory Factor 5 (IRF5) Correlates with Allograft Acute Rejection of Liver Transplantation" was retracted in 2019. Reasons: missing or withdrawn patient consent; ethical violations by an author; concerns about the data.

In conclusion, for the first time we found the genetic association between IRF5 and liver graft acute rejection. HBV infection of recipients might influence the outcome of liver graft survival, and further studies need to be performed.
